The article "Tify: A quality-based frame selection tool for improving the output of unstable biomedical imaging" was published in 2019. Journal: PLoS One.

# Tify: A quality-based frame selection tool for improving the output of unstable biomedical imaging

**DOI:** 10.1371/journal.pone.0213162

**Published:** 2019-03-11

**Authors:** Dean Philip John Kavanagh, Meurig Thomas Gallagher, Neena Kalia

**Affiliations:** 1 Microcirculation Research Group, Institute of Cardiovascular Sciences, College of Medical and Dental Sciences, University of Birmingham, Edgbaston, Birmingham, United Kingdom; 2 School of Mathematics, University of Birmingham, Edgbaston, Birmingham, United Kingdom; University of Alabama at Birmingham School of Medicine, UNITED STATES

## Abstract

The ability to image biological tissues is critical to our understanding of a range of systems and processes. In the case of *in situ* living tissue, such imaging is hampered by the innate mechanical properties of the tissue. In many cases, this provides challenges in how to process large amounts of image data which may contain aberrations from movement. Generally, current tools require the provision of reference images and are unable to maintain temporal correlations within an image set. Here, we describe a tool–Tify–which can accurately predict a numerical quality score versus human scoring and can analyse image sets in a manner that allows the maintenance of temporal relationships. The tool uses regression-based techniques to link image statistics to image quality based on user provided scores from a sample of images. Scores calculated by the software correlate strongly with the scores provided by human users. We identified that, in most cases, the software requires users to score between 20–30 frames in order to be able to accurately calculate the remaining images. Importantly, our results suggest that the software can use coefficients generated from consolidated image sets to process images without the need for additional manual scoring. Finally, the tool is able to use a frame windowing technique to identify the highest quality frame from a moving window, thus retaining macro-chronological connections between frames. In summary, Tify is able to successfully predict the quality of images in an image set based on a small number of sample scores provided by end-users. This software has the potential to improve the effectiveness of biological imaging techniques where motion artefacts, even in the presence of stabilisation, pose a significant problem.

## Introduction

The microcirculation is the primary site of gas and nutrient exchange and also provides the means for the trafficking of various cellular effectors to tissues upon demand. Upon infection, or other deleterious stimuli, circulating inflammatory cells firstly adhere to microvessels and then migrate through them towards damaged areas. Understanding these adhesive events is critical to managing diseases of the microcirculation. Fluorescent intravital microscopy (IVM) is an effective experimental tool allowing visualisation of various microvascular beds *in vivo* [1–6]. However, due to their anatomical location or normal physiological function, some tissues are in a state of constant movement which creates a significant barrier to imaging. Indeed, the beating nature, and close anatomical proximity to the respiratory movement of the lungs, has meant *in vivo* imaging of the heart has remained challenging and elusive. To minimize motion artefacts, several stabilisation techniques have been designed that physically constrain the tissue [1–3]. However, although the heart can be held still by attaching a tissue stabiliser, contraction of the myocardium itself within the window of the stabiliser cannot be fully eliminated. Recent advances in microscope and camera technology have allowed investigators to capture dynamic events at increasingly faster frame rates in such organs. However, the data generated are normally larger, with poor quality and out-of-focus frames interspersed throughout the recorded set. As a result, these data sets consist of both visually usable/stable and unusable/unstable frames. While the capture of stable frames allows for analysis of cell trafficking and recruitment, the inclusion of unstable and out-of-focus frames in the video cause problems in both processing and analysis from these data sets.

The article "Tify: A quality-based frame selection tool for improving the output of unstable biomedical imaging" was published in 2019. Journal: PLoS One.

Although it is possible to process large image datasets manually and remove poor quality frames, this is laborious and time-consuming particularly in cases where the frame count may be in the thousands. There are a number of software tools which can be used to manage image stacks containing unfavourable frames [4–9]. The vast majority of available tools are designed to compensate for image tearing/shearing that occurs following tissue movement in raster scanning image modes. This effect is seen when the tissue movement is faster than the frame rate and therefore movement artefacts are incorporated into each image frame. Few tools are designed to identify entire frames which are of a poor standard from a larger image stack. The tools that do exist rely on the user identifying reference frame(s) against which the software screens the image stack. The decisions made are mostly binary which can result in loss of data as a result of inflexibility in the frame selection process. Furthermore, they generally do make reference to, or utilise, the fundamental underlying image characteristics in each frame. This is of importance in fluorescent biomedical imaging. For instance, fluorescently labelled circulating blood cells appear as multiple bright objects against a dark background when observed using intravital microscopy. Between frames, differences in their number and location can be expected. While this means that different frames within the same capture may visually appear very different, the underlying characteristics of the image (such as the cell and background intensity) remain the same.

The article "Tify: A quality-based frame selection tool for improving the output of unstable biomedical imaging" was published in 2019. Journal: PLoS One.

In addition, these tools often require the user to select a new reference frame from each image stack for calculations to be performed against, thus limiting automation. It would be advantageous for the development of a method that can assess image quality based on the underlying image characteristics. This lends itself better to automation, which may be useful in processing data sets consisting of many stacks which themselves consist of many image frames. Using such a method, where the quality of image is related to its characteristics, would make it easier for the software to assess new image stacks that it had not previously seen. Current frame removal solutions do not consider the impact of this process on the chronological characteristics of the resulting sequence. In an image stack derived from a video, each frame is related to the others by time. If frames are removed from the stack based on quality alone and with no consideration for their position, it is possible that the processed stack may end up with large chronological gaps between frames. Thus, a method that also allows for frame selection (i.e. identifying the best frame from a range) based on quality would be advantageous.

In this manuscript, we describe Tify, a software package developed to assist users with frame rejection and selection from large image stacks. In contrast to reference frame comparison, this tool utilises multiple linear regression to identify the association between image statistics and manually provided image scores. The correlation coefficients from the regression calculation are then used to calculate a quality score for the remaining images. These coefficients can be saved and then applied to other similar image sets. Once image quality has been estimated, the software is able to remove frames below a specified cut-off value. In addition to frame removal, this software is able to operate in a frame selection mode which allows users to select the best frame from a given rolling window, meaning images can be selected while still retaining a chronological link (in other words, generating an image set which still maintains some degree of consistent time separation). In conclusion, Tify is a software tool for the processing of biomedical videos (or image stacks) generated through unstable intravital imaging. Importantly, Tify is not limited to images acquired intravitally as it can easily be applied to other imaging modalities where image variability is present.

The article "Tify: A quality-based frame selection tool for improving the output of unstable biomedical imaging" was published in 2019. Journal: PLoS One.

## Methods

### Overview

An overview of the flow of Tify is shown in Fig 1A.

**Fig 1:** Operational model of Tify. (A) Typical operation of Tify follows a clear flow-based pattern that differentiates based on user requirements.

### Image parameters

Summary image parameters are used in linear regression calculations to identify correlations and subsequently enable the software to predict image quality. Although the software was initially developed for the processing of time lapse images from the beating mouse heart, we have included a range of image statistics that may have use in other imaging models. The software uses statistics derived from each image, the majority of which are calculated by standard and well-established methods. The software, using the individual pixel grey values as a population, identifies: unique grey values (amongst the per image population of pixels), mean pixel grey value, maximum pixel grey value, population standard deviation, population skewness (Fisher-Pearson co-efficient), population kurtosis, pixel entropy, sum pixel integrated density, sum of squares, sum pixel ramp, and segment intensity deviation. Except the latter two statistics, the image statistics are calculated by the ImageMagick library during image import; the methods for these calculations are available from the source code of the project [10].

The two additional custom statistics included within the software are specifically designed to be useful in the analysis of intravital imaging. Segment intensity deviation (referred to as SID) is a measurement of the variability (standard deviation) of sum intensities across the image when split into segments. In some imaging modalities, particularly intravital imaging, one would expect each area of the image to have broadly similar intensity. If the image intensity is variable across the surface of the image, whether that be because the image is out of focus or any another reason–the variability in the intensities from each segment would increase. A value of zero would suggest perfectly uniform image intensity between segments and therefore, across the image. A sample image is provided, where we have artificially removed some elements from each corner (by cloning the background) in order to show the effect on SID (Fig 2A; top).

**Fig 2:** Methodology of SID and sum pixel ramp. (A) (i) SID is a measure of the variation of intensities across an image. As an example, in the provided panels, we have progressively cleared the image corner-by-corner to show the effect that this has on the SID value for the image. Images which have relatively uniform intensity values tend to have lower SID values. Sum intensities for each segment are shown on the image in grey. (ii) The method for calculating Sum Pixel Ramp is shown for a row of six counted pixels. The absolute difference between subsequent pixels is shown in the example calculation and the relation to Sum Pixel Ramp is shown on the right. In order to speed up processing, the software adopts a technique termed pixel stepping; rather than sample every single pixel in a row, the software samples every *n*^*th*^ pixel (e.g. each yellow dot on the example image is a sampled pixel at a pixel step of 3). (B) Changing the pixel step value changes the population statistics for SID and Sum Pixel Ramp. (i and iv) As these values are determined by calculations on absolute and summative values, an increase in pixel step reduces the total pixel count used to derive these values and tends towards a reducing in the mean value for these statistics. (ii and v) In order to keep image statistics consistent and independent of the pixel step value, the software is able to normalise these values to the total number of pixels in an image. In this instance, increasing pixel step does not significantly alter the population means. (iii and vi) Both sum pixel ramp and SID are useful indicators of image quality. We calculated the correlation coefficients between the human score provided for each image and the values for either sum pixel ramp or SID. While SID was useful for some sets and some users, we found sum pixel ramp to be highly correlated with image quality in almost all cases.

The article "Tify: A quality-based frame selection tool for improving the output of unstable biomedical imaging" was published in 2019. Journal: PLoS One.

Sum pixel ramp is the summation of the increase or decrease in pixel intensity at point (*x*,*y)*, relative to the intensity at (*x*,*y-p)* where *p* is a user-defined pixel step (default at 3) (Fig 2A; bottom). Sum pixel ramp takes advantage of the interface between intense objects and background; cells, for instance, have a clear intensity interface at their edge. When an image is blurry, the sharpness of this interface decreases. As a result, in these images, the differences in pixel intensity are lower between adjacent pixels. In order to keep these comparisons within the bounds of the image, the starting *y* pixel coordinate for sum pixel ramp and SID assessment is *y+p*.

Both custom statistics provide an option to utilise pixel stepping for speed. For instance, if loading a large image set, it may be overly laborious to calculate these custom statistics using information from every pixel in the image. For example, in these instances, it may be preferable to take, perhaps, every other pixel and to skip the interleaving pixels (example shown in Fig 2A, bottom). If the images are bigger still, it may be preferable to perform these calculations on every third pixel. In the software, we have included this as a feature referred to as *Pixel Step*. The size of the pixel step represents how many pixels are skipped when sampling for the sum pixel ramp and SID calculations. For instance, a pixel step of 10 means that every 10^th^ pixel is sampled for the generation of these statistics (the step is applied in both the *x* and *y* dimensions). Pixel stepping is only applied to the generation of the sum pixel ramp and SID statistics. Examples of the results of these statistics are shown in Fig 2B(i) and 2B(iv).

The article "Tify: A quality-based frame selection tool for improving the output of unstable biomedical imaging" was published in 2019. Journal: PLoS One.

Given that these statistics use summative values in their calculation, changing the pixel step shifts the resulting image statistics and should be considered when setting up a data set (values from an example image set are presented in Fig 2B, upper panels). However, in order to keep values consistent between preparations, an option is available in the software to normalise these statistics to the total number of pixels surveyed (values from an example image set with normalisation are presented in Fig 2B(i) and 2B(ii)). Normalising these statistics to the total number of pixels removes the differences observed as a result of changing the pixel step (Fig 2B, lower panels).

In order to identify if Sum Pixel Ramp and SID are useful in stratifying image quality, we calculated the correlation coefficient between these image statistics and the scores provided by users. Sum Pixel Ramp appeared to be well correlated to human scoring in our image sets, which high correlation coefficients for most image sets (Fig 2C(iii)). In contrast, the correlation coefficients between human scoring and SID values varied significantly between image sets being useful for some, but not others (Fig 2C(vi)).

### Multiple linear regression

Users provide Tify with manual quality scores for a small subset of image frames. Image statistics are calculated and, along with the corresponding user scores, are exported to an external statistics package, PSPP (https://www.gnu.org/software/pspp). Multiple linear regression (MLR) is then performed by PSPP, with the image statistics provided as explanatory variables and the image quality score as the dependent variable. The statistics included for each calculation are either a) decided by the user or b) decided by the software using stepwise regression techniques. The tool subsequently obtains the coefficients, their significance and the adjusted R^2^ value for the model. If running in automated mode, Tify removes variables using backward elimination based on the p-values for each component and the adjusted R^2^ for the entire model. During each round, the variable with the highest p-value (above 0.05) is removed until the adjusted R^2^ falls following a round of removal–in this instance, the variable is returned to the regression to calculate coefficients and the process ends. If no variables are left, then the stepwise process fails and user intervention is required. Although the automated MLR process is provided for user assistance, it is not proposed to be used without some degree of user oversight.

The article "Tify: A quality-based frame selection tool for improving the output of unstable biomedical imaging" was published in 2019. Journal: PLoS One.

For testing, seven users were recruited to manually score three sets of intravital images. Each image set consisted of 200 frames. All users were provided with a full description of the study, what their scores would be used for, and how we would process their data. All users participated with consent. Users were presented with image frames and asked to provide a score for each frame. Users were given information surrounding the purpose of the experiment (e.g. to identify cellular trafficking) and what information we were seeking to obtain from the images (in the example given, cellular trafficking, we were seeking full fields of view with stained cells present). We provided no other guidance in the categorisation of images except to clarify that users were free to use the scale system (0–5) in any way they sought appropriate. At the end of the analysis, the data provided by the user was saved and anonymised. Subsequently, using diagnostic options within the software, we provided the application with the manual scores from the first *n* frames from each data set (*n = 14–62*). Subsequently, we performed an automated stepwise linear regression to calculate coefficients. Using these coefficients, we subsequently calculated image scores for all images in the set. Image scores were calculated according to

$$y_{i}=\beta_{0}+\beta_{1}X_{i1}+\beta_{2}X_{i2}+\ldots .+\beta_{n}X_{in}$$

where *y*_*i*_ is the calculated score for image *i*, *β*_0_ is the calculated intercept for the model, *β*_1..n_ is the regression coefficient for the relevant parameter, and *X*_*1*..*n*_ is the value for parameter in the image *i*. These calculated scores were then compared to the human assigned scores and the correlation coefficient of these values was calculated. Two correlation coefficients were calculated, both with and without images which had been used to generate the coefficients (e.g. using images whose statistics were not used in the regression). In addition, we sought to identify the modulus distance between calculated and provided scores. This was calculated as

$$d_{i}=|S_{i^{p}}-S_{i^{c}}|,$$

where *d* represents the distance, $S_{i^{p}}$ represents the provided score for an image *i*, and $S_{i^{c}}$ represents the calculated score for a given image *i*.

The article "Tify: A quality-based frame selection tool for improving the output of unstable biomedical imaging" was published in 2019. Journal: PLoS One.

In addition, we sought to identify if consolidating statistics from multiple image sets improved the accuracy of Tify in relation to quality scoring. The statistics and scores from the first 20 frames from each set were exported for each user and combined together to form a consolidated data set. We then used this data file to run a stepwise multiple linear regression as previously described and the coefficients from this run were saved. We then used these coefficients to calculate image quality for the image sets. The calculated scores that were obtained using the original (image specific) and consolidated coefficients were then compared to manual scores and correlation coefficients obtained. In some instances, the application of non-image specific coefficient values (i.e. consolidated values from other images) resulted in calculated quality scores which correlated strongly with human scoring but were range-shifted. By way of example, a set of images may have calculated quality scores in the range of 18 to 34, but still be functionally useful (i.e. 18 represents poor images, 34 represents good images). In order to make these values useable, we have created a function within the software which normalises these scores in the 0–5 range. To do this, each value in the image set is modified as follows:

$$C_{adj}=\frac{C_{i}-C_{min}}{C_{max}-C_{min}}\times 5$$

where C_i_ is the original image score, C_min_ is the smallest image score in the set, C_max_ is the largest score in the image set, and C_adj_ is the resulting adjusted image score.

The strength of correlations were described using the determinations suggested by Evans[11]. For absolute correlation values, the following descriptors were applied: .00-.19: “very weak”, .20-.39: “weak”, .40-.59: “moderate”, .60-.79: “strong”, and .80–1.0: “very strong”.

### Image statistic consolidation and analysis

In order to identify if coefficients can be used interchangeably between image sets we took two approaches. For the first approach, we calculated coefficients from 20 frames from each of Set 1, 2, and 3. We then subsequently used those coefficients to calculate image scores for the other sets (for instance, we used Set 1 to calculate predicted scores for Sets 2 and 3, used Set 2 to calculate scores for Sets 1 and 3, and used Set 3 to calculate scores for Sets 1 and 2). We calculated the correlation of each set of calculated scores with the manual scores provided by the volunteers. We then, for each set, used step-wise MLR to derive the image set coefficients using 20 frames from the actual set in question. Using this, we then calculated the image quality using coefficients specific to the image set. This allows us to identify if using coefficients from one image set is useful for calculating the scores of another.

The article "Tify: A quality-based frame selection tool for improving the output of unstable biomedical imaging" was published in 2019. Journal: PLoS One.

Secondly, we sought to identify if consolidating data together could result in coefficients which were either better than using individual sets alone. To do this, we took data from 20 frames in each image set (both statistics and the volunteered human score) and used these to generate consolidated data sets which were used to generate coefficients (e.g. 60 frames worth of data in total). Combining data from images in this fashion may allow for the identification of overarching characteristics that relate to quality in any given imaging modality, while giving less weight to elements in an image which are either artefactual or specific to an individual set. We used these coefficients (from consolidated data) to generate image quality scores. We then calculated the correlation of these scores to volunteered human scores. In order to ensure that any changes did not relate simply to the inclusion of more data points, we also compared the results from consolidated data to image specific coefficients but based on using 60 frames for calculation.

### Frame windowing

Removing frames based on quality alone could lead to a loss of the chronological relationship between frames; for instance, a large run of removed frames can leave large time gaps in the resulting output (Fig 3 and S1 Movie). In order to help to maintain chronological links between frames, whilst still optimizing output quality, Tify utilises a windowing technique that uses a stepping frame window for image selection (QA: Quality Alone, FW: Frame Windowing; Fig 3). Given a window size of *n*; the program runs through the entire image stack, breaking the stack into sections of *n* length. Within each window, Tify identifies the image with the highest calculated image quality in the window and marks this for inclusion and excludes the other frames. To assist users, if provided with a ‘target’ image score, Tify will calculate the smallest window that can be applied ensuring images meet the specified cut-off score. To do this, the software scans windows of increasing size (in increments of 1, up to 25% of the size of the image stack) until it identifies a size in which at least one of the contained images in each window meets the provided quality target. This is the minimum window size and is calculated/presented to the user any time that the cut-off slider is changed in the software.

The article "Tify: A quality-based frame selection tool for improving the output of unstable biomedical imaging" was published in 2019. Journal: PLoS One.

**Fig 3:** Hypothetical example of frame windowing. The software has two means for removing/controlling frames. In a quality alone (QA) mode, image quality is the sole deciding factor. In this instance, the black squares represent frames which were below the specific cut off value. The second mode, Frame Windowing (FW) allows the software to select images from regular windows in the image stack based on their score. The software selects the highest scoring image in each window and rejects the others. In the above example, a window width of 4 is applied across the whole stack (the grey lines represent each window’s bounds). Although this leads to unbalanced intervals between frames, this is less impactful when considered on a macro-level.

Examples of frame windowing are provided as supplementary videos; either with the same frame rate and looped (S1 Movie), or with each video stretched to cover the same chronology as each other (S2 Movie).

### Software description

Tify is written for Windows using Visual Basic.NET. Images are handled in Tify using Magick.NET, a library for providing ImageMagick functions to .NET applications. In addition to basic image handling, Magick.NET is used to obtain most of the statistics used by Tify. Magick.NET and ImageMagick are released on the Apache and ImageMagick licences respectively (both are compatible with the GPL). Linear regressions are performed by PSPP, which is available under the GNU General Public Licence. Generation of video files is achieved via the video module of the Accord Package and FFmpeg both of which are licenced under the GNU Lesser General Public Licence. The source code and installation binary is available via Github (https://github.com/kavanagh21/TifyVBNET).

### Reference images

Tify was tested using images obtained from existing intravital microscopy studies that had taken place in our laboratory[12]. C57BL/6 mice (obtained from Envigo at 8–12 weeks age) were anaesthetised using ketamine/medetomidine (100mg/kg, 10mg/kg, respectively). All experiments were performed with ethical approval from the Birmingham Animal Welfare and Ethical Review Board (AWERB) and under an active Home Office licence. Following anaesthesia, a tracheotomy was performed, and mice were ventilated with medical O_2_ and 1.5% isoflurane (Zoetis, London, UK). Next, a cannula was inserted into the left common carotid artery for the administration of conjugated antibodies and/or vascular contrast agents. To label neutrophils, mice received a bolus administration of 20μl PE-conjugated anti-Gr-1 (RB6-8C5; eBioscience, Cheshire, UK). Mice were orientated on their sides, and the heart imaged using a 3D-printed stabiliser. Images were obtained using an Olympus BX-61WI microscope (Olympus, Southend-on-Sea, UK), with a Nipkow spinning confocal (3i, USA) and Evolve camera (Photometrics, AZ, USA). Timelapse captures were digitally captured using SlideBook software (Intelligent Imaging Innovations, CO, USA) with an exposure time of 30ms. Captures were exported as qualitative 16-bit TIFF images prior to importing into Tify.

The article "Tify: A quality-based frame selection tool for improving the output of unstable biomedical imaging" was published in 2019. Journal: PLoS One.

### Statistics

Differences between groups were analysed using paired t-tests with a p value of <0.05 considered significant. Pearson Product Moment Correlation Coefficients (PPMCC) were calculated in Excel. Where bars are present on graphs, these represent mean ± standard deviation.

## Results

### Multiple linear regression of image statistics is a reliable indicator of image quality for intravital videos

To confirm the ability of the software to calculate image quality scores, we provided the software with an increasing number of manually scored source frames (sample frames) and requested the application use these to calculate quality scores for the remaining frames (for instance, if the software used 14 frames to generate coefficients, we calculated the correlation between the human scores and the calculated score for the remaining 186 frames). Correlation coefficients between human and calculated scores reached a practical plateau at between 18–22 frames, depending on the specific image set in question (e.g. average PPMCC at 20 frames for Set 2: 0.76±0.03; Fig 4A) although they did increase gradually with increasing manual score provision (62 frames: 0.86±0.02; Fig 4A). To show visually how calculated scores compared with human scores, representative XY plots are shown of the volunteers with the best (highest) and worst (lowest) correlated scores in each set (Fig 4B, six panels).

**Fig 4:** Tify can calculate image scores which correlate well with human scoring. Users were presented with data sets that contained a variety of image types from separate experiments. Each user was presented with three sets of images, with each set containing 200 frames. Correlation coefficients were calculated for each image by comparing calculated scores with human scores. The software was given an increasing number of frames to use for calculation (horizontal axis). (A) Correlation coefficients derived from the comparison of human to machine scores, excluding the frames provided to the software. Each point represents a single user, and the solid line represents the mean of these values. (B) Example XY plots are shown for the users with the highest and lowest correlation coefficients in each set. The average numerical distance between the human and computed score for each frame was calculated for images in each set. (C) The average distance from each calculated score and the human score in each set decreases as more frames are supplied for the calculation of coefficients. Each point represents results from a single user, and the solid line represents the mean of these values.

The article "Tify: A quality-based frame selection tool for improving the output of unstable biomedical imaging" was published in 2019. Journal: PLoS One.

Next, we sought to identify if the calculated image scores were close in value to the manual scores provided by volunteers. By calculating the difference between the calculated and the human scores for each frame in each set, we were able to on average how far each frame was from the score provided by the user. The scores calculated were, in practical terms, close to the scores provided by users. The average distance between calculated scores and user scores was small at similarly sized frame counts (e.g. average distance at 20 frames, Set 3: 0.53±0.03; average distance at 62 frames: 0.41±0.02; Fig 4C). Interestingly, in some cases the use of formulaic means to calculate image scores leads to the generation of scores which are outside of the numerical range in the provided samples; for instance, in some of the representative scatter plots (Fig 4B), the software calculates the scores for some image frames to be less than zero (and equally, some frames higher than 5). Using these plots, we identified poorly calculated scores (e.g. points where the calculated score clearly deviated from the human score) and reviewed these manually. In some cases, the deviations were a result of either inconsistent scoring by users. In other cases, we identified broadly similar images by appearance but with underlying statistical differences (e.g. clear images/structure, but with reduced intensity).

### Coefficients generated from consolidated image data can be used to accurately calculate image scores

For routine use, it would be useful if pre-calculated coefficients could be used on new images. This would remove the need to score frames when using image sets that are similar to those that the user may have scored previously. To test how applicable coefficients are between images, we took two approaches–firstly, we used coefficients generated from any given image set and applied them to the remaining sets. Secondly, we created a new dataset consolidating 20 frames (and manual scores) from each of the three sets of images and then calculated coefficients from this set using stepwise multiple regression. We subsequently used the model from the consolidated data set to assess the ability of these coefficients to calculate accurate scores. Although in some cases, non-specific coefficients were equally as useful in calculating image scores when compared to image specific coefficients, generally, using non-specific coefficients resulted in significantly worse correlations between calculated and human scoring (specific: 0.77±0.02, non-specific: 0.51±0.08; p<0.01; Fig 5A). Of all the comparisons, 54% generated correlation coefficients that were at least 90% in value of those generated by image specific coefficients.

The article "Tify: A quality-based frame selection tool for improving the output of unstable biomedical imaging" was published in 2019. Journal: PLoS One.

**Fig 5:** Calculating image quality scores using coefficients generated using consolidated and non-specific image data is a potentially useful approach. (A) Calculating image scores using coefficients generated from other, non-specific, image data results in a drop in average correlation coefficients. Although the overall average correlation coefficient falls, not all instances result in a drop in this value. (B) Calculating image scores using consolidated coefficients improves the accuracy with which the software is able to predict human scoring. (C) The statistical differences observed when using consolidated data sets to generate coefficients is lost when more image frames are provided to generate scores using non-consolidated data. Using 60 frames to generate the scores from non-consolidated enhances the scoring accuracy to the same level as using coefficients from consolidated data sets. (D) Example XY plots of manual vs calculated scoring before and after range adjustment. All lines for panels A, B, and C are colour coded based on whether the correlation coefficient for each set falls to by more than 10% (red), falls but no more than 10% (blue), or increases (green).

Next, we sought to identify if consolidating frames was useful in improving the accuracy of score predictions when compared to using non-consolidated coefficients. Consolidating 20 frames from each data set improves the ability of the software to accurately predict image quality when compared to scores generated using dataset-specific coefficients (generated by processing 20 frames); this is observed by a slight but significant increase in the average correlation coefficient (e.g. original set specific coefficients: 0.77±0.02, consolidated coefficients: 0.84±0.02; p<0.001; paired t-test; Fig 5B). While this increase is statistically significant, it remains likely that the functional consequence of this is relatively small given that a shift of that size is unlikely to dramatically improve the accuracy of the software in relation to predicting scores. We next sought to identify whether this improvement in accuracy simply stems from an increase in the number of frames used to generate the coefficients. To test this, we compared scores calculated using consolidated data against scores from non-consolidated data, but increased the number of frames used to generate coefficients (from 20 to 60). Increasing the number of frames used from 20 to 60 increased the accuracy of the scoring such that no statistically significant difference remained when using consolidated coefficients (e.g. non-consolidated, 60 frames: 0.71±0.01, consolidated: 0.69±0.02; Fig 5C).

The article "Tify: A quality-based frame selection tool for improving the output of unstable biomedical imaging" was published in 2019. Journal: PLoS One.

While using coefficients generated with consolidated data, we identified that these values were significantly range shifted (examples given in Fig 5D, top panels). We built a feature into the software to automatically adjust these calculated values to bring them into the standard 0–5 range (for forward compatibility against other images) (Fig 5D, lower panels).

## Discussion

Intravital microscopy has become an invaluable tool for the monitoring of events in the microcirculation. While some tissues lend themselves well to intravital imaging[13–15], others have proven more difficult to image. In most cases, this is due to issues concerning access, motion and stabilisation. For instance, the lungs and heart have both proven difficult to image due to their anatomical location and respiratory / contractile movements (this is also a common problem for other non-intravital imaging techniques[16]). While novel stabilisation techniques have alleviated some of the problems caused by tissue motion, in most cases these techniques do not fully abolish motion artefacts. Although it is possible to synchronise imaging with physiological triggers (e.g. ECG or respiratory gating[3]), this technology is not available to all laboratories. In these instances, post-hoc image analysis is preferable. Post-hoc image analysis primarily consists of the rejection of frames which do not contribute to analysis (e.g. blurred, out of focus) and the registration of images which are subject to small motion artefacts. In this manuscript, we describe one such post-hoc processing tool which we have named *Tify*. This package is able to assign scores to image frames based on their calculated quality, on the basis that the user provides a small amount of input data (manual quality score) which can be associated with image statistics using multiple linear regression. The resultant scores can then be used to exclude or include images based on their calculated quality scores.

Several other packages exist which perform frame rejection on image stacks. This software does not supersede these, but rather provides an alternative approach for researchers to perform post-hoc frame rejection. This solution has several useful characteristics; firstly, the calculation of a quality score allows an end-user the flexibility to decide the exact point at which frames should be rejected, and to view the result in real-time. This is important, for instance, in cases where the end-user wishes to carefully balance the number of frames retained against the net quality of the resulting collection. In addition, frame windowing allows users to select frames to form the best quality time-lapse, while still enforcing a chronological linkage. During routine use, the package reports to the end-user the minimum achievable frame width based on quality cut-off settings, although users can select any window size and the software will simply select the best image from each window. Although Frame Windowing is a useful feature, it is dependent on a high enough frequency of good quality images and minimal long runs of poor images; in these situations, the software has no choice but to include poor quality images if the window width is low. In addition to these features, the formulaic nature of the software scoring process allows users to use coefficients generated from consolidated data (e.g. with data from multiple different image sets). Although it is possible to use coefficients from one image set on another, this–on average–reduced the accuracy when compared to using coefficients that were specific to each image. With that said, this does not mean that using coefficients from other image sets is never viable; in over half of cases, doing so resulted in accuracy comparable with using non-specific coefficients. It is likely that using coefficients from other image sets would need to be considered on a case-by-case basis. Finally, the software is able to consolidate statistics from numerous image stacks, allowing it to better ‘learn’ the characteristics that make up images of a certain type; such consolidation would allow users to perform frame selection without having to provide any manual scores.

The article "Tify: A quality-based frame selection tool for improving the output of unstable biomedical imaging" was published in 2019. Journal: PLoS One.

When used in automated mode, the software uses a stepwise linear regression process to arrive at coefficients to allow for the calculation of quality scores. To do this, the software performs multiple linear regression, starting with all variables (except those specifically excluded by the operator). At each stage, the routine removes the variable with the highest p-value until either a) removal of the variable reduces the adjusted R^2^ for the model or b) no non-significant variables remain. There are several potential pitfalls with stepwise regression, and particularly when lacking human intervention. In particular, the software has no prior understanding of the relevance of a particular variable from an experimental viewpoint. For instance, if an experimental setup always results in higher quality images having higher mean intensities, there is no way for the software to know this when performing the stepwise regression (although it would be highly likely that such key variables would be included in the resulting model). Without this prior knowledge, the method adopted in this software is vulnerable to multicollinearity which may result in rejection of important variables, overfitting and type II errors in respect to redundant variables[17]. It is therefore preferable that the end-user would manually consider the variables that make up the final model. In our hands, stepwise regression results in favourable results as identified by the software’s ability to accurately calculate quality for any given source image. While we would advise caution in the use of stepwise regression without interaction, our results suggest that this technique is useful in the context of this package.

Perhaps unsurprisingly, providing more data for regression analysis (in the form of manual quality scoring) results in more accurate quality scores. In most cases, the software is able to accurately calculate image quality scores after between 18–22 frames have been counted from each set. At this point, the correlation coefficients of human vs calculated scores do not improve significantly regardless of how many addition human scores are added into the model. Similarly, the average distance (how far each point is from the human score) also–broadly speaking–approaches a functional plateau at frame counts in the 20–30 range. This suggests that somewhere in the 20–30 range may be sufficient for reliable image scoring using this software. It is interesting to note that in some instances, even providing as few as 14 frames results in correlation coefficients that would be considered moderate to strong using the interpretation of Pearson’s r in Evans[11].

With Tify we have aimed to create a functional tool to enable the high-throughput scoring of imaging datasets. While this manuscript has focussed on the swift processing of these large image stacks, there is the option for sacrificing some of the speed for improvements to the accuracy of the fitting. Some of the image characteristics used in Tify’s classification are not orthogonal, adding a transformation step to orthogonalize the variables may provide a more rigorous fitting procedure. Further extensions could involve incorporating a learning database for Tify, enabling the manual correction of mis-classified images to be fed back in to future analyses, providing a more robust scoring as more data sets are analysed. Tify is an open source project, allowing interested parties to contribute to future improvements, and to modify the project to suit individual needs.

The article "Tify: A quality-based frame selection tool for improving the output of unstable biomedical imaging" was published in 2019. Journal: PLoS One.

In summary, Tify is able to successfully predict the quality of images in an image set based on a small number of sample scores provided by end-users. This then allows Tify to exclude frames based on a user-defined quality cut-off and to generate output with increased usefulness to researchers. This software has the potential to improve the effectiveness of intravital imaging techniques where motion artefacts, even in the presence of stabilisation, pose a significant problem.

## Supporting information

S1 Movie Example outputs from frame windowing, without time stretching. The top left video represents the original input to the application. The various other segments provide examples of the results from frame windowing. All videos have the same frame rate, with the videos with larger windows set to loop at the end.
(MP4)

S2 Movie Example outputs from frame windowing, with time stretching. The top left video represents the original input to the application. The various other segments provide examples of the results from frame windowing. However, in this video each of the videos has been adjusted so that they are synchronised in relation to real-time.
(MP4)
